# Effects of Chengqi Decoction on Complications and Prognosis of Patients with Pneumonia-Derived Sepsis: Retrospective Cohort Study

**DOI:** 10.1155/2021/8475727

**Published:** 2021-10-29

**Authors:** Zhipeng Huang, Xiaoxin Cai, Yao Lin, Bojun Zheng, Li Jian, Yu Yi, Yang Guang

**Affiliations:** ^1^Dongguan Hospital of Integrated Chinese and Western Medicine Affiliated to Guangzhou University of Traditional Chinese Medicine, Dongguan 523000, Guangdong, China; ^2^Guangzhou University of Traditional Chinese Medicine, Guangzhou 510405, Guangdong, China; ^3^Department of Critical Care Medicine, The Second Affiliated Hospital of Guangzhou University of Traditional Chinese Medicine, Guangzhou 510006, Guangdong, China

## Abstract

**Purpose:**

A specific and efficacious method for treatment of pneumonia-derived sepsis is lacking. Chengqi decoction has been used for treatment of pneumonia-derived sepsis, but a clinical trial on patients with pneumonia-derived sepsis is lacking, a gap in the literature that we sought to fill. *Patients and Methods*. 282 patients with pneumonia-derived sepsis admitted to the intensive care unit of our hospital were selected. They were divided into the treatment group (141 cases) and control group (141 cases). Both groups underwent conventional treatment, but Chengqi decoction (in the form of enema) was given to the treatment group. Mortality, morbidity (abdominal distension and gastrointestinal bleeding), duration of antibiotic use, and use of vasoactive agents were documented 28 days after the drug was used.

**Results:**

The treatment group reduced mortality and morbidity (abdominal distension) (*P* < 0.05). After adjustment for significant covariates, 28-day survival was similar for the whole group (hazard ratio (HR): 0.48; 95% confidence interval (CI): 0.23–0.97; *P*=0.037), for the subgroup (*n* = 120) with Acute Physiology and Chronic Health Evaluation II score ≥25 (HR: 0.180; 95% CI: 0.032–0.332; *P*=0.039) and for the subgroup (*n* = 66) with N-terminal B-type natriuretic peptide <1800 (0.059, 0.004–0.979, and 0.019). There was no difference between the two groups for the duration of antibiotic use, major bleeding, or use of vasoactive drugs.

**Conclusions:**

Chengqi decoction improved 28-day survival and reduced the prevalence of abdominal distension in patients with pneumonia-derived sepsis.

## 1. Introduction

Sepsis is a clinical syndrome involving physiological, biological, and biochemical abnormalities and life-threatening organ dysfunction caused by a dysregulated inflammatory response to infection. Sepsis and septic shock are major healthcare problems [1]. Sepsis is considered a time-sensitive emergency because the best chance for a patient to survive is to be treated promptly [2]. However, the therapeutic effect of sepsis is not satisfactory, and the mortality rate is high [3].

Severe pneumonia is caused by infection by pathogenic microorganisms and is the main infection site of sepsis [4]. Unfortunately, patients suffering from severe sepsis often develop intestinal injury, which hampers treatment [5]. Therefore, exploration of any method that can cure both pneumonia and intestinal injury is rational and urgent.

Traditional Chinese medicine (TCM) theory dictates that diseases of the lung and those of the large intestine react with each other. The occurrence and development of sepsis is related to translocation of bacterial/endotoxins in the intestines [6, 7]. However, enemas containing TCM formulations have important roles in the immunomodulation of sepsis [8].

“Chengqi decoction” (CD) is a well-known TCM formulation used commonly in China. CD has an anti-inflammatory role in sepsis and prevents translocation of intestinal flora. TCM theory also states “Fei he da chang”—“the lung and the large intestine being interior-exteriorly related” [9]. If intestinal failure occurs, a large volume of toxins accumulates in the intestinal tract, so using enemas containing TCM formulations could become a new method of sepsis treatment [10].

We wished to ascertain if CD can be used to reduce the risk of death from pneumonia-derived sepsis (PDS), abdominal distension, gastrointestinal bleeding, use of vasoactive drugs, and duration of antibiotic use. We also sought to identify the characteristics of CD that could reduce the risk of death from PDS by 28 days by relieving gastrointestinal complications.

## 2. Patients and Materials

### 2.1. Study Design

We conducted a retrospective, observational cohort study and reported its results in accordance with Strengthening the Reporting of Observational Studies in Epidemiology (STROBE) guidelines [11].

### 2.2. Study Setting and Population

This study was conducted in a 15-bed intensive care unit (ICU) at a university-affiliated tertiary-care hospital. Patients admitted to the ICU between March 2014 and September 2019 were evaluated for study inclusion. For all patients, the characteristics documented at baseline were age, sex, weight, height, body mass index (BMI), diagnosis upon hospital admission, Sequential Organ Failure Assessment (SOFA) score, Acute Physiology and Chronic Health Evaluation II (APACHE II) score, heart rate, systolic blood pressure, diastolic blood pressure, mean arterial pressure, central venous pressure, white blood cell count, neutrophilic granulocyte percentage, pH, arterial partial pressure of oxygen (PaO_2_), arterial partial pressure of carbon dioxide (PaCO_2_), PaO_2_/fraction of inspired oxygen (FiO_2_), central (mixed) venous oxygen saturation (ScvO_2_), as well as levels of lactate, N-terminal B-type natriuretic peptide (NT-proBNP), creatinine, blood urea nitrogen (BUN), C-reactive protein, and procalcitonin.

Patients (male or female) were aged >18 years. Patients were restricted to those with proven infections, defined as a positive blood culture or positive bronchoalveolar lavage fluid (BALF) culture and SOFA score ≥2; within 24 h of time, the culture was ordered [12]. Cultures positive for common contaminants (e.g., coagulase-negative staphylococci in one of two blood culture bottles and *Candida* species in BALF cultures) were excluded.

The control group comprised sepsis patients who had been in the ICU >7 days. Patients were excluded from the control group if they had a malignant tumor and advanced cachexia, had a tendency for severe bleeding or coagulation disorder, were pregnant or lactating, were infection of other systems, such as the urinary system and digestive tract infection, and had contraindications such as acute abdomen and severe cardiovascular diseases.

### 2.3. Variables

Mortality at 28 days was documented. “Abdominal distension” was defined as abdominal pressure >12 mmHg [13]. “Gastrointestinal bleeding” was defined as occult blood in feces or succus gastricus after exclusion of hemorrhoids or oral bleeding. The duration of antibiotic treatment and use of vasoactive agents were also documented.

### 2.4. Treatment

Conventional treatment (e.g., infection prevention, organ function support, resuscitation after shock, correction of disturbances in water and electrolyte balance, and maintenance of acid-base balance) and a lung-protective ventilation strategy (if necessary) were conducted for patients in both groups. On that basis, enema therapy using CD was added in the treatment group.

*Rheum officinale*, mirabilite, lobster sauce, Fructus Aurantii Immaturus, and *Magnolia officinalis* were the basic prescriptions for CD, with addition or subtraction of components as needed. Then, 200 mL of CD was fried strongly at 37°C. Enema containing CD was given once a day over 7 days.

### 2.5. Statistical Analyses

Patients were monitored after enrollment to 28 days or until death. Baseline characteristics were assessed within 24 h before enrollment. Data were analyzed using SPSS 25.0 (IBM, Armonk, NY, USA). Differences between the treatment group and control group were tested by analysis of an unpaired *t*-test, Wilcoxon's rank-sum test, *x*^2^ test, or Fisher's exact test, as appropriate. Values are the mean ± SD. *P* < 0.05 was considered significant.

Univariate Cox regression was used to model the odds of 28-day mortality. For categorical variables, HRs reflected the increased odds of 28-day mortality for absence of the variables. For continuous variables, HRs reflected the increased odds of 28-day mortality for a one-unit increase in the baseline variable. The meaningful factors of single-factor analysis were introduced into the Cox multiple regression model. Factor screening was based on gradual introduction of a removal method to calculate the HR. In addition, we undertook multivariate Cox regression analysis to model the odds of 28-day mortality using the APACHE II score, NT-proBNP level, age, lactate level, PaO_2_/FiO_2_, ScvO_2_, gastrointestinal bleeding, abdominal distension, and BMI as independent variables. A multivariate model using the APACHE II score, NT-proBNP level, and age was also used for analyses. Multivariate models reported HRs adjusted for all variables in the model. *P* < 0.05 was considered significant for all comparisons.

## 3. Results

141 patients were enrolled in the CD group, and other 141 pneumonia-suffering patients were enrolled as controls. The characteristics of the two groups of patients at baseline are given in Table 1. The groups were well-matched, except for BMI (*P* < 0.01), heart rate (*P*=0.01), procalcitonin level (*P* < 0.01), FiO_2_/PaO_2_ (*P*=0.02), ScvO_2_% (*P* < 0.01), NT-proBNP level (*P* < 0.01), and BUN level (*P* < 0.01) in the treatment group versus the control group.

Data for primary and secondary outcomes are given in Table 2. By day 28, the treatment group had a significant reduction in mortality (34.37% vs. 65.63%; *P*=0.03) and prevalence of abdominal distension (36.36% vs. 63.64%; *P*=0.02), as well as a nonsignificant increase in the prevalence of gastrointestinal bleeding (56.25% vs. 43.75%; *P*=0.58). However, there was a nonsignificant reduction in use of vasoactive agents (46.67% vs. 53.53%; *P*=0.39) and a nonsignificant decrease in duration of antibiotic use (13.23 ± 5.32 vs. 12.6 ± 5.23; *P*=0.33).

The number of cases in our study was relatively small, so the survival rate at a given time could not be calculated, and Kaplan–Meier analysis was used. There was a significant difference in survival at 28 days between the two groups (Figure 1). Survival of the treatment group was significantly higher than that in the control group. The log-rank test was also carried out and also revealed a significant difference between the two groups (*P*=0.04).

We studied the sum populations to determine the risk factors for death in each group. We applied univariate analysis of 10 potential risk factors with mortality as the dependent variable to each group (Figure 2), and the results are given in Table 3. We chose to include groups, the APACHE II score, NT-proBNP level, and age in the multivariate model (Figure 3). After adjustment by univariable analysis, one covariate was found to be significant in the multivariate analysis, and the CD group showed a HR of 0.48 (95% confidence interval (CI): 0.23–0.97; *P*=0.04).

Subgroup analyses for the HR of death at days 28 are given in Table 4. In the subgroup with an APACHE II score ≥25, the HR for probability of survival at 28 days was 0.18 (95% CI: 0.03–1.02; *P*=0.04). In the subgroup with NT-proBNP <1800 npg/mL, the HR for the probability of survival at 28 days was 0.06 (95% CI: 0.01–0.98; *P*=0.02).

## 4. Discussion

In recent years, understanding of sepsis and septic shock has gone from the tissue level to cellular and molecular levels, that is, from the theory of microcirculatory ischemia and hypoxia to the current theory of excessive release of inflammatory factors. Some scholars believe that the displacement of toxins is due to severe trauma, infection, shock, sepsis, and septic shock after surgery [14]. The pathogenesis and treatment of sepsis have been studied deeply [15, 16], but the incidence of sepsis and septic shock has not improved considerably. PDS remains a challenge in extracorporeal circuits for drug delivery in critically ill patients, and the mortality in this patient population is high [17]. However, TCM has obvious advantages over Western medicine in PDS treatment and conforms to the theory of treating pulmonary diseases through intestinal administration of drugs. Giving sepsis patients enema containing the CD formulation, combined with conventional treatment, could elicit the advantages of TCM and Western medicine [18, 19].

This was the first retrospective cohort trial investigating the effects of a 7-day course of CD treatment in patients with PDS. In this study, we chose to include groups, the APACHE II score, NT-proBNP level, and age which were filtered through single-factor analysis in the multivariate model. Meanwhile, we found that groups was the most important influencing factor, so we further analyzed the 28-day mortality between the CD group and control group. CD treatment relieved abdominal distension and led to a significant decrease in 28-day mortality. CD treatment did not increase the prevalence of gastrointestinal bleeding, duration of antibiotic use, or use of vasoactive agents. There was a significant decrease in 28-day mortality between the two groups, especially in the subgroup with an APACHE II score ≥25 and NT-proBNP <1800 pg/mL.

We demonstrated, through a retrospective cohort study, that CD could reduce 28-day mortality in patients with PDS. Improvement in the prognosis of patients with sepsis by CD has been demonstrated by several scholars [20–23]. In 2016, Mao et al. published a study on the effects of Xuan Bai Chengqi decoction (XCD) on lung compliance for patients with acute respiratory distress syndrome (ARDS). In that study, CD not only improved static compliance and dynamic compliance but also shortened the duration of parenteral nutrition and reduced the prevalence of complications and death [20]. CD also has a significant curative effect in severe pancreatitis, acute cholangitis, and myocardial ischemia [21–23].

Subgroup analyses revealed that patients with an APACHE II score ≥25 and NT-proBNP <1800 pg/mL were pronounced. These observations indicated that CD improved the prognosis of patients with PDS more significantly in the group with severe illness. In patients with good cardiac function, the effect of CD on the prognosis of patients with pneumonia and sepsis was more obvious and may have been associated with the increase of additional fluid in Chengqi decoction enema [24].

We found that CD could reduce the abdominal pressure of patients. This may have been related to the therapeutic characteristics of TCM formulations, which have multiple pathways, targets, and links. For example, Dachengqi decoction has been shown to be efficacious in ARDS treatment. Scholars have shown significant differences in the recovery time of intestinal sounds, anal exhaust time, regression of abdominal distension, as well as improvement in MODS and recovery time between two groups, indicating that Dachengqi decoction could improve the organ function of patients suffering from multiple-organ dysfunction syndrome [25–27]. Some scholars believe that TCM formulations have a good therapeutic effect on PDS and that they may act through the gastrointestinal tract. They have postulated that rhubarb can inhibit the activity of nitric oxide and inducible nitric oxide synthase to inhibit granulocyte aggregation and reduce free-radical production [28, 29]. Our study showed that CD may improve PDS through reduction of intraabdominal pressure without increasing the risk of gastrointestinal bleeding. The reduction in intraabdominal pressure may have been due to a reduction in the intestinal inflammatory response by CD.

Our study had three main limitations. First, it was conducted at a single institution. Second, the study cohort was small. Last, there was a potential selection bias to this retrospective study. Therefore, more prospective studies with larger cohorts are needed to support our findings.

## 5. Conclusion

In PDS, early administration of an enema containing CD for 7 days was safe and associated with improved survival without a significant increase in the risk of hemorrhage within the gastrointestinal tract. Our study was underpowered for an exploratory analysis to demonstrate survival benefit in patients with severe illness and good cardiac function.

## Figures and Tables

**Figure 1:** Kaplan–Meier estimate of survival on day 28 after adjustment by Cox regression analysis for the NT-proBNP level, age, and APACHE II score. The red line corresponds to the control group. The blue line corresponds to the Chengqi decoction group. The HR for probability of survival at 28 days was 0.48 (95% CI: 0.23–0.97; *P*=0.037).

**Figure 2:** Univariate analysis of 10 potential risk factors for mortality as the dependent variable to each group.

**Figure 3:** Multivariate analysis of four potential risk factors for mortality as the dependent variable to each group.

**Table 1:** Patient characteristics at baseline.

	Total	Chengqi decoction	Control	*P*
Patients (*n*)	282	141	141	—
Male (*n* (%))	162 (100)	75 (46.29)	87 (53.70)	0.223
Age (years)	67.00 (67.00–87.25)	67.00 (48.00–87.00)	67.00 (55.00–90.00)	0.484
BMI (kg/m^2^)	23.66 (21.25–25.39)	24.22 (22.04–30.48)	23.31 (20.29–25.39)	0.006
APACHE II score	24.30 ± 7.20	25.23 ± 6.33	23.40 ± 8.00	0.222
SOFA score	12.00 (11.00–15.00)	13.00 (11.00–15.00)	12.00 (10.00–14.00)	0.189
HR (bpm)	94.00 (78.00–113.25)	88.00 (60.00–102.00)	97.00 (89.00–115.00)	0.010
SBP (mmHg)	115.00 (105.00–127.50)	115.00 (105.00–126.00)	111.00 (98.00–129.00)	0.803
DBP (mmHg)	49.50 (45.00–62.25)	50.00 (44.00–63.00)	49.00 (45.00–61.00)	0.771
MAP (mmHg)	72.00 (63.00–85.50)	72.00 (62.00–83.00)	72.00 (65.00–88.00)	0.688
CVP (mmHg)	8.95 ± 5.13	8.62 ± 5.52	8.28 ± 4.61	0.204
WBC	12.56 (4.19–23.90)	4.37 (3.72–23.90)	14.19 (7.19–23.90)	0.065
NG%	81.20 (80.10–87.68)	81.20 (79.10–87.30)	81.20 (80.10–89.90)	0.655
CRP (mg/L)	73.00 (45.75–85.00)	73.00 (34.00–89.00)	74.00 (54.00–84.00)	0.303
Procalcitonin (ng/mL)	5.11 (2.50–12.30)	3.12 (1.60–7.30)	8.10 (4.50–23.90)	≤0.001
PH	7.39 (7.30–7.44)	7.38 (7.29–7.43)	7.39 (7.30–7.46)	0.137
PaO_2_	102.00 (91.00–126.00)	102.00 (91.00–126.00)	108.00 (90.40–126.00)	0.955
PaCO_2_	46.90 (44.00–60.40)	45.80 (41.50–59.10)	46.90 (44.50–61.00)	0.101
PaO_2_/FiO_2_	232.77 ± 64.61	217.58 ± 63.68	247.95 ± 62.14	0.021
Lactate (mmol/L)	1.95 (1.30–3.30)	1.79 (1.30–2.60)	2.10 (1.30–4.00)	0.246
ScvO_2_	64.31 ± 13.81	59.86 ± 13.79	68.69 ± 12.35	0.002
NT-proBNP (pg/mL)	5348.50 (2201.00–12180.00)	2392.00 (1569.00–7810.00)	7899.00 (3883.00–15015.00)	≤0.001
SCr (*µ*mol/L)	184.39 (97.16–280.80)	113.39 (95.34–280.00)	188.00 (154.90–308.00)	0.106
BUN (mmol/L)	13.19 (8.80–16.41)	10.50 (7.58–15.20)	15.61 (12.00–19.66)	≤0.001

SOFA, sequential organ failure assessment; BMI, body mass index; APACHE, Acute Physiology and Chronic Health Evaluation; BUN, blood urea nitrogen; HR, heart rate; SBP, systolic blood pressure; DBP, diastolic blood pressure; MAP, mean arterial blood pressure; CVP, central venous pressure; WBC, white blood cell; NG%, neutrophilic granulocyte percentage; CRP, C-reactive protein; PaO_2_, arterial partial pressure of oxygen; PaCO_2_, arterial partial pressure of carbon dioxide; PaO_2_/FiO_2_, arterial partial pressure of oxygen/inspired oxygen fraction; ScvO_2_, central (mixed) venous oxygen saturation; NT-proBNP, N-terminal B-type natriuretic peptide; SCr, serum creatinine.

**Table 2:** Primary and secondary outcomes.

	Total	Chengqi decoction	Control	*P*
Primary outcome				
Mortality (*n* (%))	96 (100)	33 (34.37)	63 (65.63)	0.03

Secondary outcomes				
Abdominal distension (*n* (%))	165 (100)	60 (36.36)	105 (63.64)	0.02
Gastrointestinal bleeding (*n* (%))	48 (100)	27 (56.25)	21 (43.75)	0.583
Duration of antibiotic use (days)	12.92 ± 5.31	13.23 ± 5.32	12.6 ± 5.23	0.332
Vasoactive agent (*n* (%))	180 (100)	84 (46.67)	96 (53.53)	0.391

**Table 3:** Univariate and multivariate models for overall survival on day 28.

Covariate at study entry	HR	95% CI	*P*
Univariate models			
NT-proBNP (pg/mL) (<1800 vs. ≥1800)	0.31	0.09–1.00	0.05
BMI (kg/m^2^) (18–23 vs. >23 or <18)	1.51	0.76–3.02	0.24
Age (years) (≤65 vs. >65)	1.70	0.84–3.41	0.14
Gastrointestinal bleeding (present vs. absent)	0.67	0.23–1.90	0.44
Abdominal distension (present vs. absent)	0.73	0.36–1.46	0.37
APACHE II score (<25 vs. ≥25)	2.12	0.98–4.59	0.06
FiO_2_/PaO_2_ (<150 vs. ≥150)	0.04	0.01–13.60	0.29
Lactate (mmol/L) (<2 vs. ≥2)	0.65	0.32–1.31	0.23
ScvO_2_ (%) (<75 vs. ≥75)	0.85	0.40–1.85	0.69
Group (Chengqi decoction vs. control)	0.48	0.23–0.97	0.04

Multivariate models			
Group (Chengqi decoction vs. control)	0.48	0.23–0.97	0.04^*∗*^
APACHE II score (<25 vs. ≥25)	2.02	0.89–4.60	0.09
NT-proBNP (pg/mL) (<1800 vs. ≥1800)	0.34	0.09–1.19	0.09
Age (≤65 years vs. >65 years)	1.39	0.67–2.88	0.38

^*∗*^Adjusted for: NT-proBNP, age, APACHE II score. HR, hazard ratio; NT-proBNP, N-terminal B-type natriuretic peptide; BMI, body mass index; FiO_2_/PaO_2_, inspired oxygen fraction/arterial partial pressure of oxygen; ScvO_2_, central venous oxygen saturation; APACHE, Acute Physiology and Chronic Health Evaluation.

**Table 4:** Subgroup analyses of the risk of death in the Chengqi decoction group and control group at 28 days.

Subgroup	Chengqi decoction (*n* = 141)	Control (*n* = 141)	HR with Chengqi decoction (95% CI)	*P*
Age				
<65 years, *n*/total (%)	18/63	36/63	0.30 (0.08–1.08)	0.06
≥65 years, *n*/total (%)	15/78	27/78	0.45 (0.13–1.70)	0.21

APACHE II score				
<25, *n*/total (%)	27/78	42/84	0.53 (0.18–1.58)	0.25
≥25, *n*/total (%)	6/63	21/57	0.18 (0.03–1.02)	0.04

Lactate (mmol/L)				
<2, *n*/total (%)	15/81	24/60	0.34 (0.09–1.28)	0.10
≥2, *n*/total (%)	18/60	39/81	0.46 (0.14–1.56)	0.21

NT-proBNP (pg/mL)				
<1800, *n*/total (%)	3/54	6/12	0.06 (0.01–0.98)	0.02
≥1800, *n*/total (%)	30/87	57/129	0.67 (0.25–1.76)	0.41

HR, hazard ratio; APACHE, Acute Physiology and Chronic Health Evaluation.

## Data Availability

The data used to support the findings of this study are included within the article.
